# Health Risk Assessment of Pesticide Residues in Drinking Water of Upper Jhelum Region in Kashmir Valley-India by GC-MS/MS

**DOI:** 10.1155/2023/6802782

**Published:** 2023-01-27

**Authors:** M. Imran Ganaie, Ishrat Jan, Afshan Nabi Mayer, Alamgir A. Dar, Ishtiaq A. Mayer, Pervez Ahmed, Javid A. Sofi

**Affiliations:** ^1^Department of Geography and Disaster Management, University of Kashmir, Srinagar 190006, India; ^2^Research Centre for Residue and Quality Analysis, Sher-e-Kashmir University of Agricultural Sciences and Technology (SKUAST-K), Shalimar Campus, Srinagar 190025, India; ^3^SSM College of Engineering, Srinagar 193121, India

## Abstract

Globally growing demand for agricultural and farm foods has more or less become dependent on chemical pesticides to maintain the supply chain, which undoubtedly boosts agricultural production. However, pesticides not only impact the target pests but cause hazard to human health. Pesticides are ubiquitous and can be found in almost every component of the environment. They can therefore impair human and biota health when present over the threshold level. The present study assessed the concentration of commonly used pesticides for agricultural purposes but get mixed in different sources of water, as such fifteen sampling sites along the upper Jhelum basin of Kashmir valley were chosen. For the analysis, 60 water samples were obtained from different water sources. Gas chromatography coupled with tandem mass spectrometry (GC-MS/MS) was used to determine pesticide residues in water samples. Pesticide residues from 10 of the 26 commonly used pesticides were detected in water samples. Difenoconazole had the highest concentration among the pesticides detected, with a mean concentration of 0.412 ± 0.424 *μ*g/L ranging from 0.0 *μ*g/L to 0.8196 *μ*g/L. The target hazards quotient (THQ) was used to quantify the possible noncarcinogenic health risks associated with drinking pesticide-contaminated water. Only chlorpyrifos and quinalphos were detected >1 in RWS3 (1.6571), RWS4 (1.0285), RWS14 (1.2571), and RWS15 (1.2000) sample sites, implying that the drinking water poses a health risk to humans. Hence, pesticide hazards should be mitigated and rigorous monitoring is needed to reduce pesticide residues in drinking water.

## 1. Introduction

Pesticides are valuable interventions in modern agriculture, but the risks and benefits of using them must be carefully considered and monitored [1–3]. Crop yields and agricultural output have increased dramatically as a consequence of innovative practices such as the use of various types of pesticides and chemical fertilizers; therefore, they have become an integral part of the modern agrarian system. However, at the same time, excessive and indiscriminate use of pesticides has resulted in negative effects on human health [4–8].

Pesticides are ingested through multiple modes of exposure (inhalation, ingestion, and skin contact) from various environmental mediums (soil, water, air, and food), causing health complications to varying degrees [9–12]. As a result of their volatilization, pesticides are efficiently transported into the ground and surface water and contaminate the aquatic ecosystem through infiltration, spray drift, drainage water, runoff, leaching, and atmospheric deposition [13–15]. This may happen due to improper practices like filling of sprayers, washing of spraying equipment, discarding pesticide packages, and throwing the leftover solution into the water [13]. Water solubility, weather conditions (temperature, precipitation, and wind), soil type, and agricultural management practices are all associated with this sort of pollution [16–18]. Pesticides are more vulnerable to surface water in places where intensive agriculture and horticulture are the prevalent occupations, posing a significant threat to human water consumption. Pesticide residues in river systems pose a threat, not only to human health by consuming water but also to fish and other aquatic species [19–21].

Contamination of water is further triggered by indiscriminate use of pesticides in agriculture and horticulture by unintentional release of such hazardous substances to adjacent nontarget ecosystems viz., rivers, springs, groundwater, etc. [20]. Pesticides even at low concentrations pose a serious threat to the environment and human health [22], thereby pesticides are toxic not only to those who work in agriculture and horticulture fields but also to the general populace [23]. Various studies throughout the world notably [20, 24–28] employ target hazards quotient approaches to estimate pesticide hazards. The US Environmental Protection Agency (USEPA) conducts human health risk assessments based on some published guidelines and policies, including general principles for performing aggregate exposure and risk assessment [29], guidelines for carcinogen risk assessment [30], and exposure factors handbook [31]. Chronic pesticide exposure over a tolerable level can have negative repercussions and provide noncarcinogenic risks to people, which can be more severe in vulnerable groups including the elderly, pregnant women, and children [20, 32]. The USEPA established target hazard quotient (THQ) which is generally used to evaluate the possible noncarcinogenic human health concerns associated with long-term oral exposure to polluted water. The THQ-based risk assessment approach provides a reasonable indication of risk levels associated with pollutant exposure [33].

Almost every type of pesticide is used by fruit growers (Spray schedule, 2021). The widespread use of pesticides in apple orchards is concerning. The rapid conversion of agricultural land into orchards during the last two decades has resulted in the excessive and indiscriminate use of pesticides, the majority of which are composed of harmful chemicals such as dimethoate, chlorpyrifos, mancozeb, captan, quinalphos, dodine, fenazaquin, carbendazim, tebuconazole, flusilazole, difenoconazole, hexaconazole, and myclobutanil as depicted in Table 1 [34] (Spray schedule, 2021). Furthermore, the indiscriminate use of pesticides has polluted water bodies around these horticultural and agricultural regions. The study region is situated in an area where horticulture is the predominant commercial crop, which further contributes to the relevance of the research. Given this, the purpose of this study is to assess the pesticide residue assessment with health risks involved in drinking water of the upper Jhelum basin in Kashmir valley. Therefore, it is one of the prime issues to ensure the management of freshwater resources in the study area. The findings of this study may be used by policymakers to promote environmental pollution management, prioritize highly polluted locations in the upper Jhelum basin of Kashmir Valley, and find strategies to mitigate the negative consequences of pesticides on human health.

## 2. Materials and Methods

The commonly used pesticides in horticulture and agriculture are mentioned in Table 1. These commonly used pesticides from thirteen chemical families were assessed. Among the types of pesticides, fungicides, followed by insecticides, acaricides, herbicides, and rodenticides, are the most frequently used pesticides. Pesticides including dimethoate, chlorpyrifos, quinalphos, fenazaquin, tebuconazole, flusilazole, difenoconazole, dithianon, dodine, ziran, copper oxychloride, and thiacloprid are classified as moderately hazardous, while hexaconazole and myclobutanil come under the toxicity class of slightly hazardous and only carbofuran is classified as highly hazardous, and the rest comes under the classification of unlikely to pose an acute hazard in normal use recommended by the World Health Organization.

### 2.1. Study Area

The study area is a major part of southern portion of the Kashmir Valley. It consists of four administrative districts, namely, Anantnag, Pulwama, Shopian, and Kulgam. It forms the upper Jhelum portion of the Kashmir Valley and is located at an altitude of 1570 to 5300 meters above the mean sea level (Figure 1). It lies between 34°16′10″ and 33°21′30″N latitude and 74°30′20″ and 75°37′26″E longitude [35]. The geographical size of the study area is 5454 km^2^. The average population density in the study area is around 360 people per square kilometre. The majority of people reside in rural regions. The most prevalent economic activity is agriculture and horticulture [36]. Due to the Indian winter monsoon, which delivers western disturbances imbedded in large-scale subtropical westerlies, the study region experiences precipitation during the entire winter season [37]. The study area's average maximum and minimum temperatures are 19.27°C and 7.29°C, respectively, with 84 cm of annual rainfall. Temperatures can drop to −9°C in the winter and reach 38°C in the summer [38, 39]. The study area is surrounded by high mountains, which remain snow-clad for most of the year and are gifted with plenty of snow-fed springs, rivers with a network of their tributaries, and freshwater lakes [40]. These freshwater lakes, which come from a variety of sources such as snow-fed, spring-fed, and groundwater aquifers, provide water for drinking, irrigation, and other domestic needs. River Jhelum, the trunk stream of the Jhelum basin originates in the study area near Verinag and flows almost through the entire length of Kashmir Valley [41, 42].

Agriculture and horticulture are the most common occupations in the study region, accounting for 19.80 and 7.49 percent of land use, respectively [43]. The study area is predominantly an agricultural society with favourable agro-climatic conditions, fertile soil, and a temperate climate, which are ideal for the growing of fruits and vegetables and offer enormous potential for the development of horticultural operations in the region. The horticultural sector makes a substantial contribution to the region's economy [4]. Nature has endowed Kashmir with a rich biodiversity as well as some incredible fruit crops that are barely found in the rest of the world. People in Kashmir grow a range of cash crops such as apple, almond, walnut, cherry, and other fruits and nuts since the valley has fertile soil, a favorable climate, and natural water supply [34].

### 2.2. Chemicals

The technical grades of all the pesticide standards (purity 99.0%) were obtained from Sigma-Aldrich, India. Solvents, salts, and reagents like dichloromethane, acetone, hexane, sodium chloride (NaCl), (ASC reagent grade ≥99.9%), and analytical grade-activated anhydrous MgSO_4_ were obtained from Merck, Darmstadt, Germany. Sodium sulphate (Na_2_SO_4_) anhydrous (AR grade) was acquired from S. D. Fine Chemicals, Mumbai. All solvents were redistilled in all-glass apparatus prior to the use, and the suitability of the solvents and other chemicals was ensured by running reagent blanks before actual analysis.

### 2.3. Preparation of Standard Solution

Standard stock solutions of different pesticides (1 mg·mL^−l^) were prepared separately in HPLC grade n-hexane for GC-MS/MS analysis. For calibration curve, different concentrations (1.0, 0.75, 0.5, 0.10, 0.05, and 0.01 *μ*g mL^−1^) were prepared with appropriate dilution of the stock solution. The solutions were filtered through 0.45 *μ*m PTFE filter before analysis. All standard stock solutions and working standard solutions were stored at 4°C before use.

### 2.4. Sampling

Pesticides' influence on water quality was determined using a multistage sampling approach. From September 2020 to August 2021, water samples were taken seasonally from fifteen distinct sampling sites. The sampling sites were selected considering altitude and agricultural land use pattern, and the secondary source of data has been used for this purpose (Figure 1). Since the bulk of people in the study area use stream water, nine samples were chosen from streams and two from protected tap waters, springs, and wells, respectively. River/stream water samples were collected at sampling sites RWS1, RWS2, RWS3, RWS4, RWS5, RWS6, RWS13, RWS14, and RWS15; tap water samples were collected at sampling sites TWS11 and TWS12; spring water samples were collected at sampling sites SWS7 and SWS8, and groundwater samples were collected at sampling sites GWS9 and GWS10 (Table 2). Domestic water supplies rely heavily on water drawn from rivers and streams. The two springs were selected because they serve as a community resource, while the other groundwater and tap water test locations were chosen for comparative purposes. The population around these sampling locations is long-established orchard growers and rice cultivators, except for the samples of spring and tap water. Eleven sample locations were chosen in order to include hotspots of pollution discharges along the different streams and rivers, such as orchard and paddy field zones. Thereby, large amount of chemical pesticides are applied. However, all of these sites are interconnected to each other through streams and their tributaries. The two springs chosen for sampling are the origins of two rivers as well; one is the source of the Aripal stream and the other is the source of the main river Jhelum. Water samples were collected in high-purity two-liter glass bottles, marked with unique sample IDs, and transported in an icebox to the *Pesticide Residue analysis Laboratory, SKUAST-Kashmir, Shalimar, Srinagar,* where they were kept at 4°C until extraction. A total of 60 water samples were collected from diverse drinking water sources spread over four administrative districts (Anantnag, Kulgam, Pulwama, and Shopian) for pesticide residue analysis. The sampling approach employed in this study is similar to that used in previous related research [13, 20, 44–47].

### 2.5. Sample Preparation

A separating funnel was used to collect 750 ml of water from each sample site; it was added with 150 g of sodium chloride and was shook until it was completely dissolved. We add 100 ml dichloromethane and shake it vigorously for 1 minute by releasing pressure frequently and collect the bottom lower layer by passing through anhydrous sodium sulphate in a 500 ml conical flask [48]. The procedure was repeated for the same extraction two more times with 50 ml of dichloromethane and was collected in the same flask after passing the anhydrous sodium sulphate [49–51]. The collected layer of samples (organic phase) was dried in a rotatory evaporator and was then dissolved three times in 15 ml *n*-hexane and evaporated near to dryness, and we finally reconstituted the sample with 1 ml acetone : Hexane (1 : 9) [52–54].

### 2.6. Instruments

The cleaned extracts were analyzed on Agilent gas chromatography-mass spectrophotometer (GC-MS/MS). The separation of pesticides was done on a Capillary column: Agilent J&W HP-5 ms UI 30 m × 0.25 mm × 0.25 *μ*m. The GC parameters for analysis are as follows: The inlet was set at ∼27.5 psi (constant pressure mode) during run. Helium was used as carrier gas with the injector temperature set at 280°C. The injector was used in the split less mode. The oven was operated as follows: initially, the temperature of the oven was set at 70°C (held for 2.0 min), heated to 150°C at 25°C/min, then heated to 200°C at 3°C/min, and finally raised to 280°C at 8°C/min (held for 10.0 min). The transfer line temperature in MS was kept at 280°C. The total run time was 41.867 min; ion source temperature 300°C, and MS quadrupole temperature, 180°C. The MS system was set in the multiple reactions monitoring (MRM) mode. The LOD of all the pesticides was 0.01 mg/kg and LOQ was 0.05 mg/kg.

### 2.7. Statistical Analysis

In order to analyze the general distribution of residual pesticide concentration in water samples, descriptive statistics (mean and standard deviation) were computed. Second, the inferential statistics were performed using the Target Hazards Quotient (THQ) to evaluate any potential noncarcinogenic health effects related to drinking pesticide-contaminated water.

### 2.8. Target Hazards Quotient

The target hazard quotient (THQ) was used to assess the possible noncarcinogenic health concerns associated with drinking pesticide-contaminated water. THQ based on the methodology was used by [13, 20, 24, 25, 55].

(1) $$\begin{array}{c} THQ=\frac{\left(EF\times ED\times WIR\times C\right)}{\left(RfD\times BW\times AT\right)}\text{,} \end{array}$$

where EF = exposure frequency = 365 days/year, ED = exposure duration = 70 years (equivalent to the average human lifetime), WIR = water ingestion rate = 2000 mL/person/day, C = pesticide concentration in water (mg/L), RfD = acute reference dose [56] (Table 3), BW = body weight = 70 kg/person, and AT = average time in days = 365 days/year × ED. If the THQ value is ≥1, exposed people may experience health risks by consuming pesticide-contaminated water. As a result, actions and safeguards must be implemented.

## 3. Results and Discussion

### 3.1. Concentration of Pesticides in Water

The results of detected pesticide residues in drinking water are summarized in Table 4. Out of twenty-six commonly used pesticides, ten were detected in the diverse drinking water sources. All the sampling sites detected dimethoate, chlorpyrifos, myclobutanil, hexaconazole, and fenazaquin, except for two spring water samples SWS7 and SWS8, which were below the detection limits (BDL). Difenoconazole had the highest concentration among the pesticides detected, with a mean concentration of 0.412 ± 0.424 *μ*g/l ranged from 0.0*μ*g/l to 0.8196 *μ*g/l in the sampling site RWS6 followed by site RWS3 with 0.396 ± 0.376 ranged from 0.0 *μ*g/l to 0.7965 *μ*g/l. Both the concentrations were highest in spring season (March to May) because most of it was sprayed during these seasons. Meanwhile, all of the sites with a concentration BDL seemed to have the lowest concentration of the pesticides detected. These areas are located between 1970 and 1900 meters above the mean sea level, where the use of pesticides is almost negligible. The other sites having the concentration of BDL are those that were obtained after the treatment. Pesticide contamination was found in tap water as well but at very low concentrations. The treatment plants in the study area employ conventional treatment techniques, and these plants do not remove pesticides from water [21]. The sites with IDs RWS1, RWS2, RWS3, RWS4, RWS5, RWS6, GWS9, GWS10, RWS13, RWS14, and RWS15 were found to contain tebuconazole and flusilazole, while the rest of the sites with low concentration (BDL) were tap water and spring water samples. Except three sampling sites, namely, SWS7, SWS8 and TWS11, difenoconazole is below the detection limit. All the river/stream water sampling sites with IDs RWS1, RWS2, RWS3, RWS4, RWS5, RWS6, RWS13, RWS14, and RWS15 spiromesifen were detected, whereas the rest of the sites were BDL. At sample locations SWS7, SWS8, TWS10, and TWS11, it was found that quinalphos was below detection limit (BDL).

Pesticides were only identified in two seasons, namely, spring and summer, from March onwards to August because the bulk of pesticides in the study area are applied during these months [66, 67]. During the autumn and winter seasons, no pesticides were detected. Since contamination of surface water from agriculture and horticulture is a widespread problem, it should come as no surprise that the detection of pesticide residues was most common in this kind of water [68–71]. Due to erosion, soil from surrounding horticultural and agricultural areas may instantly enter river water, maintaining high pesticide concentrations [13, 72, 73].

### 3.2. Human Health Risk Assessment

The target hazards quotient (USEPA 1989) of the pesticides detected in the study area of the various sources of drinking water is shown in Table 5 (Figure 2). The THQ assessment was based on the average residual concentration in terms of the noncarcinogenic risks of the pesticides that were found in the water samples. Risk assessment of the pesticide residue concentration in different water sources in the study area was compared to the acute reference dose (ARfD), which is the threshold limit of health significance. Only chlorpyrifos and quinalphos were greater than 1, of the ten pesticides detected in the fifteen sample sites. The THQ value of chlorpyrifos was greater than 1 in RWS3 (1.0571) sampling site, while the THQ value of quinalphos was greater than 1 in RWS3 (1.6571), RWS4 (1.0285), RWS14 (1.2571), and RWS15 (1.2000) sample sites indicating that the drinking water of these sites poses health risks to humans. The THQ value for the remaining sites was less than 1, indicating that the health hazards posed by these substances were permissible. The sampling sites with a THQ greater than one are those surrounded by orchard fields where most of the pesticides are sprayed. Pesticide pollution is more likely to occur around agriculture and horticulture fields due to spray drift and runoff from agricultural and horticulture land transporting pesticides to nearby surface water [74–76]. Toxins from pesticides used in orchard farms and paddy fields in the research area have seeped into rivers and streams, damaging drinking water sources [77, 78]. In the study area, substantial amount of pesticides is sprayed on orchards from the spring season (March onwards) until the summer season (till August). This is the time when a variety of pesticides are sprayed on crops to protect them from preharvest to postharvest operations [79, 80]. These get washed into small rivulets and streams, ultimately reaching the Jhelum River and its tributaries. If it rains after the pesticide application, the drinking water sources become even more contaminated [77, 81]. The concentration of pesticides was higher in sampling sites near agriculture and horticulture fields than in sampling sites that are distant away. The longer distance could play a role in lowering concentration due to dilution and continued reduction of residues [13]. Anthropogenic pollution of water systems can come from a variety of sources, including chemical industry discharge [82, 83], domestic sewage [84], agricultural wastes [85–89], and residues of pesticide [90–97]. Figure 2 was generated in ArcGIS-10.3 software and depicts the distribution of detected pesticides in different sampling sites using IDW (inverse distance weighted) interpolation.

The results of the current analysis confirmed the presence of pesticides in the water; however, they were not exceeding acceptable limits. Horticulture is expanded considerably in the study region, from 3.2 percent in 1990 to 7.49 percent in 2017, thereby horticulture uses the majority of pesticides in the study area [4, 43, 98, 99], and the sector has emerged the most dominant land-use, absorbing mostly fertile agricultural land use in the non-Karewa belt [100–102]. Agriculture and horticulture are the most common activities in the study region, accounting for 19.80 percent and 7.49 percent of land usage, respectively [43]. This indicates that more pesticides are required in the future, and the pesticide concentration burden in drinking water, especially surface water, will rise. Pesticide use will become a concern for human and animal health if it grows in lockstep with the development of horticulture land use. Humans might suffer from both chronic and acute health issues. This emphasizes the significance of focusing more attention on improving farmer awareness of pesticide usage in both the aquatic and terrestrial ecosystems throughout the upper Jhelum watershed basin of the Kashmir Valley. Pesticide risks should be reduced by identifying places that are more susceptible to pesticides, particularly areas nearby sources of drinking water.

Furthermore, knowledge, attitude, and practice concerning pesticide usage and waste disposal among pesticide applicators are critical attributes to foster among farmers. Farmers' attitudes, knowledge, and behaviour towards pesticide safety can also be used to control pesticide discharge. It is strongly recommended that seminars should be held to educate farmers, urging them to obtain enough knowledge and raise awareness about the harmful effects of pesticides and promote workplace health and safety, especially in places where water bodies are nearby [4, 103].

## 4. Conclusion

In this study, the occurrence of pesticide residue with human risk assessment of twenty-six pesticides from thirteen chemical families was assessed, with five chemical families having pesticides detected. Residues in water were identified only during the spring and summer seasons, owing to pesticide application during these seasons. Contamination is found in regions dominated by agricultural and horticulture land use due to the result of various environmental causes, including leaching and seeping into nearby surface and groundwater, agricultural runoff, and spray drifts from indiscriminate pesticide application. Agriculture and horticulture are the primary sources of pesticide contamination. Water bodies in close proximity to these locations are more vulnerable than those distant away. For the health risk assessment, the average individual pesticide concentration in each sample is taken into account. Only chlorpyrifos and quinalphos have a THQ greater than 1, indicating a considerable risk of pesticide exposure. RWS3, RWS4, RWS14, and RWS15 are the four sample sites where THQ is reported more than one. All four sampling locations are in close proximity to agricultural and horticulture land use. Hence, consistent water quality monitoring has been recommended for drinking water sources in the upper Jhelum basin (South Kashmir) of the Kashmir Valley. It is suggested that pesticides should be used sustainably, and bio-pesticides should be sought as alternatives because they are less detrimental to the environment [104].

## Figures and Tables

**Figure 1:** Study area & sampling site map; source SOI toposheets 1971 & satellite data 2017.

**Figure 2:** (a) Interpolation diagrams (A and B) showing spatial distribution of detected pesticides in the study area. (b) Interpolation diagrams (C and D). (c) Interpolation diagrams (E and F). (d) Interpolation diagrams (G and H). (e) Interpolation diagrams (I and J).

**Table 1:** Commonly used pesticides in south Kashmir and their toxicological class recommended by WHO.

S.no	Registered names	Chemical class	Toxicity class	Type
1	Mancozeb	Organosulphur	U	Fungicide
2	Propineb	Dithiocarbamate	NC	Fungicide
3	Zineb	Dithiocarbamate	U	Fungicide
4	Captan	Phthalimide	U	Fungicide
5	Dodine	Aliphatic nitrogen	II	Fungicide
6	Ziram	Dithiocarbamate	II	Fungicide
7	Dithianon	Quinone	II	Fungicide
8	Hexaconazole/Myclobutanil	Triazole	III	Fungicide
9	Dimethoate	Organophosphate	II	Insecticide
10	Quinalphos/chlorpyrifos	Organothiophosphate	II	Insecticide
11	Flusilazole	Organosilicon	II	Fungicide
12	Trifloxystrobin	Strobilurin	U	Fungicide
13	Tebuconazole/difenoconazole	Triazole	II	Fungicide
14	Hexythiazox	Thiazolidine	U	Acaricide
15	Spiromesifen	Titronic acid	NC	Acaricide
16	Fenazaquin	Unclassified acaricide	II	Acaricide
17	Chlorothalonil	Organochlorine	U	Fungicide
18	Metiram	Dithiocarbamate	U	Fungicide
19	Pyraclostrobin	Strobilurin	NC	Fungicide
20	Carbendazim	Benzimidazole	U	Fungicide
21	Copper oxychloride	Copper fungicide	II	Fungicide
22	Thiacloprid	Thiazolidine	II	Insecticide
23	Carbofuran	Carbamate	Ib	Nematicide

Ib: highly hazardous; II: moderately hazardous; III: slightly hazardous; U: unlikely to pose an acute hazard in normal use; NC: not classified; source: spray schedule SKUAST-K, Department of Horticulture Kashmir & Field survey 2020 [34].

**Table 2:** Sampling sites description of south Kashmir drinking water sources.

Sampling IDs	Water sources	Sampling location	Geo-coordinates	Altitude mts (m)
RWS1	Rimbiara stream	Hirpora village	33.694930N 74.795458E	2100
RWS2	Vishav/rimbiara	Naina village	33.818030N 75.066535E	1590
RWS3	Vishav stream	Nihama village	33.633056N 74.891794E	1960
RWS4	Vishav stream	Puhloo village	33.64406N 75.05402E	1686
RWS5	Lidder/jhelum	Odur village	33.753014N 75.131277E	1610
RWS6	Jhelum river	Sangam	33.830466N 75.070121E	1580
SWS7	Verinag spring	Verinag	33.534820N 75.249587E	1970
SWS8	Aripal spring	Aripal village	34.015353N 75.069994E	1900
GWS9	Tube well	Chitragam village	33.768631N 74.973903E	1700
GWS10	Tube well	Rathsuna village	33.905337N 75.120311E	1618
TWS11	Tap water	Kakapora village	33.949508N 74.932693E	1572
TWS12	Tape water	Niloora village	33.814941N 74.984869E	1620
RWS13	Lidder stream	Seerhamdan village	33.787542N 75.230159E	1644
RWS14	RumshiNallah	Drabgam village	33.833969N 74.815273E	1632
RWS15	Aripal stream	Chandigam village	33.904091N 75.06121E	1589

RWS: river water sample; SWS: springwater sample; GWS: groundwater sample; TWS: tape water sample.

**Table 3:** Detected pesticides with ARfD and ADI values.

Detected pesticide	ARfD mg/kg BW/day	ADI mg/kg BW/day	References
Dimethoate	0.01	0.001	[20, 57, 58]
Chlorpyrifos	0.005	0.001	[20, 57, 58]
Myclobutanil	0.31	0.025	[59]
Tebuconazole	0.03	0.03	[59]
Flusilazole	0.02	0.002	[56, 60]
Difenoconazole	0.1	0.01	[56, 61]
Hexaconazole	0.03	0.005	[56, 62]
Spiromesifen	2.0	0.03	[63]
Fenazaquin	0.1	0.05	[64]
Quinalphos	0.0005	—	[65]

ARfD: acute reference dose; ADI: acceptable daily intake.

**Table 4:** Distribution of detected pesticides residues in different water sources of south Kashmir.

Detected pesticides (*μ*g/l)	*μ* ± *σ*	*μ* ± *σ*	*μ* ± *σ*	*μ* ± *σ*	*μ* ± *σ*	*μ* ± *σ*	*μ* ± *σ*	*μ* ± *σ*
*Sampling sites*	*RWS1*	*RWS2*	*RWS3*	*RWS4*	*RWS5*	*RWS6*	*SWS7*	*SWS8*
Dimethoate	0.021 ± 0.024	0.020 ± 0.023	0.103 ± 0.181	0.049 ± 0.073	0.019 ± 0.022	0.022 ± 0.026	<LOD	<LOD
Chlorpyrifos	0.018 ± 0.021	0.103 ± 0.174	0.185 ± 0.243	0.113 ± 0.163	0.095 ± 0.113	0.159 ± 0.227	<LOD	<LOD
Myclobutanil	0.035 ± 0.024	0.053 ± 0.038	0.420 ± 0.477	0.331 ± 0.370	0.041 ± 0.029	0.295 ± 0.466	<LOD	<LOD
Tebuconazole	0.102 ± 0.119	0.232 ± 0.373	0.309 ± 0.362	0.357 ± 0.412	0.396 ± 0.452	0.343 ± 0.396	<LOD	<LOD
Flusilazole	0.025 ± 0.019	0.033 ± 0.025	0.034 ± 0.026	0.033 ± 0.025	0.031 ± 0.023	0.066 ± 0.056	<LOD	<LOD
Difenoconazole	0.259 ± 0.405	0.289 ± 0.420	0.396 ± 0.376	0.261 ± 0.244	0.304 ± 0.307	0.412 ± 0.424	<LOD	<LOD
Hexaconazole	0.032 ± 0.036	0.182 ± 0.316	0.195 ± 0.323	0.180 ± 0.299	0.176 ± 0.299	0.053 ± 0.061	<LOD	<LOD
Spiromesifen	0.011 ± 0.021	0.021 ± 0.024	0.023 ± 0.027	0.024 ± 0.028	0.020 ± 0.024	0.017 ± 0.019	<LOD	<LOD
Fenazaquin	0.014 ± 0.027	0.044 ± 0.055	0.029 ± 0.033	0.027 ± 0.031	0.041 ± 0.053	0.051 ± 0.058	<LOD	<LOD
Quinalphos	0.011 ± 0.013	0.014 ± 0.021	0.029 ± 0.035	0.018 ± 0.022	0.012 ± 0.016	0.016 ± 0.021	<LOD	<LOD

*Sampling sites*	*GWS9*	*GWS10*	*TWS11*	*TWS12*	*RWS13*	*RWS14*	*RWS15*	
Dimethoate	0.010 ± 0.020	0.009 ± 0.018	0.010 ± 0.020	0.005 ± 0.010	0.051 ± 0.078	0.071 ± 0.117	0.022 ± 0.026	
Chlorpyrifos	0.019 ± 0.038	0.020 ± 0.041	0.008 ± 0.012	0.006 ± 0.010	0.017 ± 0.021	0.088 ± 0.156	0.090 ± 0.143	
Myclobutanil	0.064 ± 0.052	0.056 ± 0.042	0.001 ± 0.003	0.012 ± 0.024	0.088 ± 0.086	0.045 ± 0.031	0.107 ± 0.146	
Tebuconazole	0.037 ± 0.043	0.021 ± 0.033	<LOD	<LOD	0.176 ± 0.295	0.232 ± 0.418	0.050 ± 0.059	
Flusilazole	0.014 ± 0.025	0.014 ± 0.025	<LOD	<LOD	0.031 ± 0.025	0.032 ± 0.025	0.032 ± 0.025	
Difenoconazole	0.051 ± 0.043	0.040 ± 0.034	<LOD	0.001 ± 0.002	0.251 ± 0.363	0.362 ± 0.445	0.189 ± 0.205	
Hexaconazole	0.038 ± 0.044	0.034 ± 0.040	0.002 ± 0.003	0.001 ± 0.002	0.081 ± 0.123	0.108 ± 0.178	0.052 ± 0.068	
Spiromesifen	<LOD	<LOD	<LOD	<LOD	0.008 ± 0.017	0.007 ± 0.015	0.015 ± 0.018	
Fenazaquin	0.028 ± 0.032	0.027 ± 0.031	0.010 ± 0.020	0.010 ± 0.020	0.070 ± 0.107	0.095 ± 0.157	0.040 ± 0.050	
Quinalphos	0.013 ± 0.016	0.014 ± 0.019	<LOD	<LOD	0.017 ± 0.023	0.022 ± 0.025	0.021 ± 0.025	

*μ*: mean; *σ*: standard deviation; LOD: limit of detection.

**Table 5:** Target hazards quotient of detected pesticide residues in different water sources of south Kashmir.

Detected pesticides (*μ*g/l)	THQ	THQ	THQ	THQ	THQ	THQ	THQ	THQ
*Sampling sites*	*RWS1*	*RWS2*	*RWS3*	*RWS4*	*RWS5*	*RWS6*	*SWS7*	*SWS8*
Dimethoate	0.0600	0.0571	0.2942	0.1400	0.0542	0.0628	0.0000	0.0000
Chlorpyrifos	0.1028	0.5885	1.0571^*∗*^	0.6457	0.5428	0.9085	0.0000	0.0000
Myclobutanil	0.0032	0.0049	0.0387	0.0300	0.0038	0.0271	0.0000	0.0000
Tebuconazole	0.0971	0.2209	0.2942	0.3400	0.3771	0.3266	0.0000	0.0000
Flusilazole	0.0357	0.0471	0.0485	0.0471	0.0442	0.0942	0.0000	0.0000
Difenoconazole	0.0470	0.0825	0.1131	0.0745	0.0868	0.1177	0.0000	0.0000
Hexaconazole	0.0300	0.1733	0.1857	0.1714	0.1676	0.0504	0.0000	0.0000
Spiromesifen	0.0002	0.0003	0.0003	0.0003	0.0003	0.0002	0.0000	0.0000
Fenazaquin	0.0040	0.0125	0.0082	0.0077	0.0117	0.0165	0.0000	0.0000
Quinalphos	0.7428	0.8000	1.6571^*∗*^	1.0285^*∗*^	0.6857	0.9142	0.0000	0.0000

*Sampling sites*	*GWS9*	*GWS10*	*TWS11*	*TWS12*	*RWS13*	*RWS14*	*RWS15*	
Dimethoate	0.0285	0.0026	0.0285	0.0142	0.1457	0.2028	0.0628	
Chlorpyrifos	0.2171	0.2342	0.0457	0.0340	0.0971	0.5028	0.5142	
Myclobutanil	0.0029	0.0051	0.0001	0.0011	0.0081	0.0041	0.0098	
Tebuconazole	0.0352	0.0200	0.0000	0.0000	0.1676	0.2209	0.0476	
Flusilazole	0.0200	0.0200	0.0000	0.0000	0.0442	0.0457	0.0457	
Difenoconazole	0.0145	0.0114	0.0000	0.0003	0.0717	0.1034	0.0540	
Hexaconazole	0.0361	0.0323	0.0019	0.0010	0.0771	0.1028	0.0495	
Spiromesifen	0.0000	0.0000	0.0000	0.0000	0.0001	0.0001	0.0002	
Fenazaquin	0.0091	0.0088	0.0028	0.0028	0.0200	0.0271	0.0114	
Quinalphos	0.7428	0.0800	0.0000	0.0000	0.9714	1.2571^*∗*^	1.2000^*∗*^	

^*∗*^THQ > 1.

## Data Availability

This manuscript comprises all of the data collected and analyzed during the research. Tables and figures in the manuscript contain the data that have been utilized to support the findings.
